The article "Edge-Enabled Heart Rate Estimation from Multisensor PPG Signals" was retracted in 2023. Reasons: signs of a paper mill; compromised peer review; unreliable results or conclusions.

# Edge-Enabled Heart Rate Estimation from Multisensor PPG Signals

**DOI:** 10.1155/2023/4682760

**Published:** 2023-02-22

**Authors:** Xingchi Chen, Fa Zhu, Hai Zhao

**Affiliations:** ^1^School of Computer Science and Engineering, Northeastern University, Shenyang 110819, China; ^2^College of Information Science and Technology, Nanjing Forestry University, Nanjing 210037, China

## Abstract

Heart rate (HR) estimation from multisensor PPG signals suffers from the dilemma of inconsistent computation results, due to the prevalence of bio-artifacts (BAs). Furthermore, advancements in edge computing have shown promising results from capturing and processing diversified types of sensing signals using the devices of Internet of Medical Things (IoMT). In this paper, an edge-enabled method is proposed to estimate HRs accurately and with low latency from multisensor PPG signals captured by bilateral IoMT devices. First, we design a real-world edge network with several resource-constrained devices, divided into collection edge nodes and computing edge nodes. Second, a self-iteration RR interval calculation method, at the collection edge nodes, is proposed leveraging the inherent frequency spectrum feature of PPG signals and preliminarily eliminating the influence of BAs on HR estimation. Meanwhile, this part also reduces the volume of sent data from IoMT devices to compute edge nodes. Afterward, at the computing edge nodes, a heart rate pool with an unsupervised abnormal detection method is proposed to estimate the average HR. Experimental results show that the proposed method outperforms traditional approaches which rely on a single PPG signal, attaining better results in terms of the consistency and accuracy for HR estimation. Furthermore, at the designed edge network, our proposed method processes a 30 s PPG signal to obtain an HR, consuming only 4.24 s of computation time. Hence, the proposed method is of significant value for the low-latency applications in the field of IoMT healthcare and fitness management.

## 1. Introduction

Heart rate (HR) estimation has been embedded into numerous portable physiological monitoring terminals, such as Internet of Medical Things (IoMT) devices [1], body area network (BAN) devices [2], wearable devices [3], remote video devices [4], and even smartphones [5, 6]. Because of the technological advance of high-performance PPG optical sensors over the years, the PPG technique is employed by more and more IoMT health and wearable devices to monitor our body status. The reason for its dominance is that the built-in PPG sensor in a device can conveniently measure the changes in the blood volume of epidermal tissues. The acquired waveform represents a PPG signal, which superimposes a variety of physiological components, such as HR, respiration, oxygen saturation [5], nervous activity, and thermoregulation. Among them, the HR estimation using a low-cost IoMT device is a most intuitional and useful method to understand our cardiovascular activity status and the pathological state of various heart diseases since the periodicity of a PPG signal is synchronized with that of cardiac rhythm. Knowledge of HR component would provide a wealth of clinical and healthy information.

However, HR estimation, even at a resting or relative stability state, using a PPG signal collected by single sensor is vulnerable to the biological artifacts (BAs). It always transpires because of various factors, including the autonomic regulation of the peripheral circulation, arterial and venous blood flow, and neurological and cardiovascular diseases. More notably, despite the introduction of multisensor PPG signals can facilitate the solution to these problems to a certain extent, data computing and sharing in the current cloud-based computing model cannot adapt to the requirements of low-latency and high-performance HR estimation from multisensors.

Edge computing, as an emerging computing paradigm, provides an innovative opportunity for the synchronized computing of multisensor PPG signals in the proximity of the edge networks. Advancements in edge computing have the desired computing capacities for the rapid development of Internet of Things (IoT) [1], Internet of Vehicles (IoV) [7, 8], Satellite-Terrestrial Networks [9], reconfigurable wireless communications [10], and video streaming processing [11–14], especially in IoMT. The explosive proliferation of IoMT generates massive amounts of time-series data, such as PPG signals. In the meantime, these data demand low-latency processing and analysis at the edge of networks not be transmitted to the centralized cloud servers. On the contrary, the addition of edge computing offers a feasible computing platform support for the computing boundary condition and low-latency requirement during resolving the BAs.

Cardiovascular system asymmetry (CSA) is a natural feature in the regular cardiovascular system [15]. This asymmetry reflects a significant property in the structure of the blood vessel system. However, the CSA provides a good basis for the generation of the BAs. Not only does it have a high chance of contaminating PPG signals but it also brings inconsistent biological noise into double-sided blood vessels. Those random vasculopathies (such as thrombus and atherosclerosis) and blood vessel variation can directly give rise to the emergence of the BAs, which means that bilateral blood vessels exist in the distribution of inconsistent biological artifacts. If the arterial compliance of bilateral vascular is inconsistent significantly, the BAs become strong. The PPG signals collected from different sensors comprise a diverse range of biological artifact components, which severely corrupt the morphological feature of PPG signals.

Biological artifacts (BAs) are a considerable barrier for HR estimation using a single PPG signal from single sensor. Since the cardiovascular system of a person is a closed-loop whole, the sampling of any PPG signal by one sensor just reflects one aspect of the overall system, that leads to the creation of the BAs. The BAs may be derived from bilateral blood vessels branches. The pathological change of vascular function based on physiological causes, e.g., atherosclerosis, vascular tumor, and arteritis, can cause some irregular changes for the light path of a PPG signal in the human tissue. In the case of vasculopathies, two important vascular characteristics, for example, dicrotic notch and diastolic peak [16], may vanish thoroughly in the time domain.

As shown in Figure 1, this is a typical example of the BAs for a person. In the left branch of the cardiovascular system, there is a certain vascular disease in his left arm, resulting in the presence of a poor PPG signal quality. In contrast, the right arm is normal, and the corresponding PPG signal is better in morphology. Apparently, there is a difference between the amplitude of two PPG signals. The amplitude of left PPG signals ranges from 100 to 200 and that of right PPG signals ranges from 80 to 300, approximately. Meanwhile, the left PPG signals have a morphological loss. In contrast, the right PPG signals are relatively intact. These are non-negligible influences for HR calculation based on PPG signals, especially for the processing of multisensor and multichannel PPG signals. If a conventional fixed threshold method is used to compute HR in this case, different HR results are attained with a high probability. In this situation, the two results of HR estimation computed separately from bilateral arterial branches may generate serious inconsistencies, e.g., the HR value measured by the left arm is 80 bpm and the other side HR maybe 65 bpm. These two HR results are from the same person and computed by the same type of devices and algorithms, which is a typical example caused by the emergence of BAs.

Recently, HR estimation from PPG signals is a hot topic in the fields of IoMT and smart healthcare [17–20], due to the convenient acquisition and pivotal physiological implications of PPG signals. In real life, the PPG signals measured from various IoMT devices are not perfect waveform. Wrist-based measurement of PPG signals is subject to the interference from some noise sources. The low-quality PPG signals can lead to the inaccuracies of HR detection and even affect diagnosis results. A challenging problem with HR estimation is the technique of artifact removal from the captured PPG signals. Especially under intense exercise conditions, many constructive approaches have been published. Most of them focus on measuring HR from intense motion-contaminated PPG signals [21–27], but also some of them calculate other physiological information, such as interbeat interval (IBI) [19], oxygen saturation (SpO_2_) [19, 22, 24], and beat-to-beat (RR interval) [25]. Not that, in this article, the *P* peak of PPG signals is equivalent to the *R*-peak in the ECG signals; that is, the representation of RR interval replaces that of PP interval. So far lately, the signal filter method is one of the most popular techniques, such as spectral masking approach (SMA) [18], least mean squares (LMS) [19], recursive least squares (RLS) [21], and multiple reference adaptive noise cancellation (MRANC) [23]. A high-performance HR estimate approach not only needs to overcome various artifacts superposed on PPG signals but also the differential representation of the models to the PPG signals.

In the condition of small magnitude motion or motion-free, the BAs should be paid attention in PPG signals. As a matter of fact, the PPG signals from different body parts are homologous signals, and all PPG signals are derived from the heart via different transmission paths. The homologous signals generate conspicuous signal drifting after different transmission paths, so that the PPG signals superimpose different artifact components. Experimental study [28] has demonstrated that the amplitude and variability of the PPG signals collected using green-light (525 nm) sensor vary greatly at different measurement sites, including the lateral and medial upper arm, lateral and medial forearm, lateral and medial wrist, and ring finger. Most of the existing approaches ignore this point and randomly capture PPG signals from single sensor. In many practical situations, particularly for clinical and fitness application, the BAs are inevitable when performing the HR estimation with the PPG sensors. Fortunately, the multisensor PPG technique can hardness more useful HR-related information and help us to distinguish the BA components from the acquired multisensor PPG signals.

In addition, many advanced techniques [29–31] have been applied in the field of IoMT and edge computing, and these techniques promote the development and innovation of processing physiological signals, especially for PPG signals. For example, the technology stack of machine learning [32–34] has greatly improved the detection and inferring capabilities of related diseases benchmarked against physiological signals and medical data. Advanced signal processing techniques [35–37] also provide a powerful reference for the processing of these medical data, especially multichannel or array signals. Most of the IoMT tasks, e.g., HR estimation, are delay-sensitive applications, and generate the data that would be timely processed on the resource-constrained edge devices. The low-latency processing of multisensor PPG signals is a challenge to the traditional cloud computing-based computing model. In the contrary, the addition of edge computing offers a feasible computing platform support for the computing boundary condition and low-latency requirement during resolving the BAs.

In order to avoid the impact of the BAs, we introduce multisensor PPG signals from bilateral blood vessels to deal with this problem. The bilateral PPG signals in both wrists are applied to support a multisensor PPG technique. Consequently, there are several challenges and difficulties to be solved in this paper. (1) The BAs are an inevitable phenomenon for an adult and is a map of the CSA. Due to the presence of the BAs, it increases the probability that an undesired PPG signal is selected. It is a challenge for working out this problem. (2) Due to the use of multisensor PPG signals, it can increase the complexity of the peak distribution for the used signals. Moreover, individual independence of testers exacerbates this problem and then results in increasing the difficulty of accurate RR interval calculation. The RR interval is a significant precondition for HR estimate in the time domain. Hence, it is a challenge to detect RR interval under the condition of using synchronously multisensor PPG signals. (3) Although the multisensor PPG signals based on bilateral blood vessels can deal with the BAs, this approach enlarges the computing volume of the PPG data. The computing paradigm based on cloud servers do not have the capacity of providing low-latency response for real-time multiple PPG signals, which is a bottleneck due to its centralized architecture. So, how to implement a low-latency and stable heart rate estimation using multisensor PPG signals on realistic low-cost edge devices is also a new challenge.

To solve the abovementioned challenges, we propose an edge-enable method to calculate HR from multisensor PPG signals. Our major contributions are summarized into three folds:

- We establish a real-world edge network using four resource-constrained edge devices to support HR estimation by multisensor PPG signals. According to this network scheme, an edge computing strategy is designed, which divides edge nodes into collection nodes and computing nodes. This strategy reduces the transmitted volume of PPG signals, improving the speed of HR computing. This scheme provides the computing platform and strategy of low-latency and high-performance for the application of HR estimation.
- In view of this edge computing platform, we present an edge-enabled heart rate estimation approach via multisensor PPG signals. As a first step in reducing the impact of BAs, we propose a self-iteration RR interval calculation to adapt the sophisticated peak distribution of multisensor PPG signals. Then, we give the detailed mathematical derivation for this portion. In order to further reduce the impact of BAs on HR estimation, while overcoming the problem of limited bounds of HR estimation brought by setting a global threshold, we establish a heart rate pool (HRP), while using an unsupervised outlier-detection method to obliterate abnormal instantaneous heart rate (IHR) from the HRP and recovering useful HR data.
- We build a dataset with multisensor PPG signals and ECG signals for illustrating the performance of our proposed method. A series of comprehensive experiments on this dataset demonstrate that our proposed method achieve excellent performance in views of the robustness, accuracy, and computing time.

## 2. Related Work

Although the PPG technique is very popular and convenient, it is highly sensitive to the artifacts caused by multifarious reasons. The artifacts reported in reference [38] can be divided into three aspects: (1) device artifacts (e.g., power interference); (2) extrinsic artifacts, including various motion artifacts; and (3) intrinsic artifacts caused by physiological reasons, for instance, cardiovascular system asymmetry (CSA) [15]. Two main hurdles for HR detection are extrinsic and intrinsic artifacts, corresponding to motion artifacts and biological artifacts, respectively. These artifacts seriously hamper the use of PPG in activities of physiological parameters detection, particularly HR estimation. A large number of studies have attempted to harness single sensor and multisensor PPG techniques to remove artifacts from PPG signals to attain an accurate HR. So, we illustrate the existing works for HR estimation by the single-sensor PPG technique, multisensor PPG technique, and motion artifacts removal technique of PPG signals.

### 2.1. Single-Sensor PPG Technique for HR Estimation

Single-senor PPG technique means that the PPG sensor is integrated in an individual chip module, providing cardiac rhythm information for HR estimation through a single PPG signal. A single-sensor PPG signal (if the SpO_2_ is computed needing two PPG signals with different wavelengths of PPG) is leveraged to estimate HR [17–19, 21, 24]. However, these categories usually need a complicated filter algorithm [18, 19, 21, 24] to extract HR-related component from a single PPG corrupted by intensive motion artifacts. Meanwhile, these algorithms require specific reference signals to be used together, for example, the acceleration signals and ECG signals. Although these HR estimation strategies are very effective under some certain conditions, they rely heavily on the use of reference signals. Once the reference signal is corrupted or the frequency spectrum of motion artifacts severely overlaps with that of HR component [24], these techniques fail to reduce the motion artifacts effectively in the most applications. It would be difficult to get an accurate and stable HR estimate in the condition of incomplete artifact reduction.

Just only collecting PPG signals from one sensor, the HR estimation is unreliable once most of them are invalid severely. These illustrate that a single sensor PPG signal as measuring signal source is limited to the capacity of expression. If the essence of signal source is defective, these methods above are invalid. Single-sensor PPG signals are infeasible in many real-world situations, for cardiovascular system monitoring and physiological measurements.

### 2.2. Multisensor PPG Technique for HR Estimation

Multisensor PPG technique consists of multiple PPG sensors, which either come from the same integrated chip (i.e., multichannel PPG sensors) or from multiple separate chips. Multisensor PPG signals as one of the multisensor PPG technique, especially for synchronous bilateral PPG signals [16, 39], are able to express more useful information of the cardiovascular system [40, 41], reducing the impact of the BAs on HR estimation.

Some authors have tried to solve the relevant cardiovascular challenge by using a multisensor PPG technique, in particular for multisensor PPG signals. The multisensor PPG signals indicate that the acquired PPG signals have a certain physical interval, and each PPG signals can characterize specific physiological components of the same cardiovascular system. Multisensor PPG signals are not necessarily multiple PPG signals obtained from the same sampling area and are possibly from different sampling regions. The blood circulatory system is one part of the cardiovascular system, whose structure, in general, is almost symmetrical. The PPG signals captured from different body parts have differentiation [28], albeit for a healthy person. In one side of the body, Maria et al. [41] has verified that there are some different characteristics in the morphology and frequency spectrums of the ear, thumb, and toe PPG signals. Furthermore, Wu et al. [16] utilized the different features of bilateral PPG signals to recognize peripheral arterial stenosis. Some clinical studies, though, have shown that in left and right arms, there usually exists an interarm systolic blood pressure difference [42]. A great discrepancy of interarm blood pressure (more than 10 points) may increase the likelihood of cardiovascular threat risk. In terms of extracting HR, these research studies have provided strong pieces of evidence that measuring bilateral blood vessels includes more enough physiological information than measurements of a one-sided blood vessel.

To extract HR parameter, these techniques fuse multiple signals, e.g., ECG, ABP, BCG, and different wavelengths PPG or multichannel PPG array. Since the ECG, ABP, and BCG can reflect identical HR information directly, C. H. Antink et al. [43] combined these three signals to extract the HR. In reference [26], Nathan and Jafari leveraged a generalized particle filter to track HR information in the emergence of motion artifacts. The ECG signals affected by noise and the PPG signals corrupted by motion are fused and introduced into particle filter to extract the HR component. In comparison of these reports, the method of Warren et al. [27] presents another way to compute HR. Two pairs of red and IR LEDs are utilized to enhance the light intensity. Among the four LEDs, six photodetectors are deployed. Multiple photodetectors are used instead of a single detector. This design can enhance the light intense received by photodetectors and improve the performance of PPG signals. As already noted, it is a crucial precondition, for HR estimation, that whether we can accurately detect the HR-related peak. In most practices, lots of interference are induced into the PPG signals so that we cannot directly measure accurate HR. So, multisensor PPG signals should be paid more attention, due to more useful and alternative HR-related information being provided.

### 2.3. Artifacts Removal Technique of PPG Signals

As one of the territories of PPG signal processing, removing artifacts, particularly motion artifacts, has received lots of attention in the past years, from 2015 to 2021. Both academia and industry have invested a large amount of human and scientific resources into the motion artifacts removal of PPG signals. Many popular techniques of artifacts removal in several influential journals are summarized in Table 1. Most algorithms of HR estimation mentioned in the table have been published in some top journals and conferences. The performance of the HR algorithm is related to many factors, such as the wavelength of PPG sensors, PPG sensor quantity and deployment area, the number of PPG sampling sensors, artifact type, algorithm type, the required additional reference sensor, and other biological signals. Among these factors, PPG sensor quantity, PPG sensor deployment area, and the use of threshold in HR estimation are the three primary determinants.

1. For the number of PPG sensors, several researchers have illustrated that an accurate HR can be calculated from a single PPG signal in different sensors [17–19, 21, 24, 44]. These methods which use a single PPG signal rely heavily on other signals (e.g., accelerometer, multiple PPG signals, BCG signals, ECG signals, and ABP signals) to provide complementary information. By various technologies of filtering and spectral analysis, motion artifact components can be successfully separated from the raw PPG signals. Furthermore, some scholars [19–21, 27] have noticed that a single PPG signal lacks sufficient references for PPG signals denoising, so that multiple PPG signals are introduced to accomplish the duty of motion artifacts removal and an acceptable result of HR estimation has been obtained. As summarized in Table 1, all algorithms capture PPG signals from one body sensor, in which 2 to 9 PPG sensors are used [19–21, 27]. To sum up, increasing the number of PPG sensors can improve the reliability of the HR components and indeed has a certain effect on HR estimation.
2. The deployment area of PPG sensors also plays an important role in accurately estimating HR. In practice, PPG signals from diverse deployment areas reveal the distribution feature of harmonic components. In some existing literatures, by combining with more information from different auxiliary signals, some studies reduce the influence of motion artifacts from PPG signals and have yielded a good result of HR computation in the diverse sampling sensors of the body, for example, wrist [17, 18, 20, 21, 23, 26], finger [22, 24], back [25], forehead [19, 22, 27], and palm. For sampling from the same area, the correlation between multiple PPG signals is relatively high. The collected PPG matrix contains a large amount of redundant information. Due to the sophisticated structure of the CSA, a poor sensor placement may introduce an adverse effect on the HR estimate. In this case, it is difficult to collect a high-quality PPG signal as a signal source, so that the problem of insufficient effective information of PPG signals can only be solved by aggrandizing the complexity of the algorithms.
3. As well-known, a suitable threshold is of great importance for the HR estimation in accuracy and robustness. Regardless of using the time or frequency domain method, a less controversial approach is to comprehensively determine the optimal threshold for extracting the main HR component in PPG signals after multiple experiments. However, in this situation, the optimal threshold is usually set to a fixed empirical or experimental value, and then, the choice of threshold determines the accuracy and robustness of the HR algorithm. These fixed thresholds cannot be adaptively adjusted for different PPG signals and ensure the accuracy of the HR estimate. Moreover, some of the reported research studies [4, 17–22, 27, 43, 44] (see Table 1) both utilize several fixed thresholds to identify the HR components from PPG signals. Due to the existence of the CAS, the collected PPG signals from different body sides and parts contain several differentiated physiological noise components. These fixed thresholds hinder an accurate calculation of physiological arguments, resulting in the poor robustness of the algorithm.

In addition, as shown in Table 1, some scholars have also tried to tune the HR results by changing the PPG sensor wavelength (e.g., 570 nm [20], 660 nm [19], and 940 nm [22]) and algorithm type (e.g., various filtering techniques [19], spectrum decomposition [17], matrix calculation [20], and time-frequency spectral analysis [22]) as well as introducing more auxiliary signals. The raw PPG signals with significant motion artifacts can be considered as a collection of desired PPG signals and motion interference signals. The filter technique can reduce motion artifacts by subtracting the accelerometer signals from PPG signals [18]. In reference [17], the JOSS method is proposed to compute HR from PPG signals corrupted by strong motion artifacts. By using synchronous accelerometer signals, the JOSS mainly is leveraged to assess the frequency spectrum information of PPG instead of using initial methods, such as spectral masking approach (SMA) [18], least mean squares (LMS) [19], and time-frequency spectral features [22]. By employing the signal decomposition capabilities of SVD, the literature separates the pure PPG signals from the corrupted PPG signals [20]. A motion artifact detection algorithm is proposed by using the time-frequency spectral information of PPG signals [22]. This algorithm is capable of detecting the corrupted PPG segments and eliminating the unusable data segment from the corrupted PPG signals. It can be seen that all works in Table 1 focus on several cardiovascular activities monitoring, such as HR, AHR, IBI, and S_*p*_*O*_2_. These parameters of health are derived from the PPG signals, and the number of PPG ranges from 1 to 9. However, most methods [17–19, 21, 27, 44] listed in Table 1 need an accelerometer signal as the auxiliary or reference signal to compute physiological parameters from the motion-corrupted PPG signals. In many clinical and life scenarios, some commercial pulse oximeters and IoMT devices do not have the support of the accelerometer; whereas, more notably, all these publications only aim at removing motion artifacts from PPG signals but cannot pay attention to the impacts of biological artifacts on the HR calculation.

To sum up, the components of HR and artifacts are real in a raw PPG signal. The proportion of motion artifacts in the collected PPG signals significantly rises as the scenario of the PPG collection is moved from a stationary state into a nonsteady state. For instance, from the clinic to the fitness or other real-world environments, the movement of application scenario results in an imperfect separation between the PPG-related and motion-related components. Due to the representation of the motion signature by the acceleration signals, it can be approximatively regarded as an estimation of the motion artifact components, and thus, the previous algorithms can utilize this property to subtract the motion artifact components from the recorded PPG signals. However, for the stationary state, BAs are the crucial issue that should be solved, not the motion artifacts. The reason, incidence, and morphology of artifacts vary significantly among individuals [38]. Different from removing motion artifacts, the accelerometer signals cannot be used as an approximate representation of the BAs. Therefore, in the next section, we discuss multisensor PPG signals and edge computing to remove the BAs.

## 3. The Proposed Method

In this section, several components of our proposed approach are introduced, totally 4 stages, such as the edge network, preprocessing, self-iteration RR interval calculation, heart rate pool, and abnormal IHR removal. In our approach, we gradually improve the performance of our algorithm by Section 3 and Section 2. Our major goal here is to remove the impact of the BAs for HR estimate, while keeping an accurate and low-latency average HR estimation based on two IoMT sensors and three resource-constrained edge devices.

### 3.1. Overview of the Proposed Method

HR measurement conducted with bilateral PPG signals exhibits the differences arising from nonuniform distribution muscle, artery-clogging, atherosclerosis, peripheral artery disease, and other cardiovascular variations or physiological structure problems. Therefore, different HR calculation results can be found using multisensor PPG signals. If we chose only one-side wrist vessel to collect the PPG signals at random, we cannot obtain the most accurate of the real HR estimate. We instead place two PPG sensors in the left and right wrist areas to facilitate HR estimation.

In this paper, we propose an edge-enabled heart rate estimation approach (EeHRA) based on multisensor PPG signals, as shown in Figure 2. In this approach, two types of edge nodes, e.g., collection edge nodes and computing edge nodes, are used to execute the task of HR estimation. As shown in Figure 2, there are four stages in our proposed method. The first stage is just for the basic procedure and a preprocessing stage which uses DB5 wavelet transform to remove power interference and baseline wander (see Section 3.3). The next is the self-adaptive RR interval calculation stage (see Section 3.4). This stage is used to carry out RR interval measurement adopting different distributions of peaks from multisensor PPG signals. In the next stage, the EeHRA leverages time domain RR intervals to compute the IHRs. A heart rate pool (HRP) is established via the IHRs calculated from both wrists' PPG signals and using an unsupervised outlier-detection method to remove the abnormal IHRs from the HRP (see Section 3.5). Finally, the average HR is estimated using the data remaining in the HRP (see Section 3.6).

### 3.2. Edge Network

In this section, we design and implement a real-world edge network with four resource-constrained devices.  Figure 3 refers to the edge network. The network composition and computing strategy are described as follows.

In this network, as shown in Figure 3, there are four parts such as IoMT devices, collection edge nodes, gateway, and computing edge nodes. For the IoMT devices, two PPG sensors (MAX30112 and Maxim Integrated Products, Inc.) and one ECG sensor (BMD101, NeuroSky, Inc) are used; the sampling rate of the PPG sensor is 200 Hz; ECG sensor has a sampling rate of 512 Hz. The collection edge nodes are composed of three resource-constrained devices whose types are Raspberry Pi 4B with 4G RAM and Quad core Cortex-A72 (ARM v8) 64 bit SoC @ 1.5 GHz. The computing edge node consists of a Raspberry Pi 4. For the gateway, the router is the TP-LINK WAR1200L with a 1200 Mbps wireless transmission rate and a wireless network support frequency of 2.4 G or 5 G.

In addition, we design a special computing strategy for this network scheme. In the collection edge nodes, we perform the functions of preprocessing and RR interval calculation. For the computing nodes, other parts of our proposed method run on this type of edge nodes and compute the final average HR. This process compresses the data volume of the collected PPG signals to less than 10%. This design effectively compresses the transmitted volume of PPG signals and provides the ability of low-latency HR estimation.

### 3.3. Preprocessing

In this paper, the preprocessing consists of two parts: (1) time calibration and calculation turn-on judgment of the PPG signals and (2) remove basic noise including the baseline wander and power frequency interference in the raw PPG signals, so as to reduce the difficulty of RR interval calculation.

#### 3.3.1. Time Calibration

Time calibration has two functions: one is to confirm whether the two PPG signals are synchronized and the other is to determine whether the execution turn-on condition of the heart rate estimation method is satisfied. Since each PPG sensor communicates with an independent collection edge node, our proposed method, in seconds (s), inserts two timestamps (start and end) for each collected PPG signal to calibrate time of multiple PPG signals.

Let timestamp_start(*τ*)_soc_ and timestamp_end(*λ*)_soc_, ∀*τ*, *λ* ∈ [1, *ε*] represent a start and end of PPG signal, respectively. If soc=1, it means that timestamp_start(*τ*) and timestamp_end(*λ*) belong to the PPG signals derived from the left PPG sensor. Similarly, if soc=2, these two parameters come from the right PPG sensor. The parameter *ε* should satisfy the following equation:

(1) $$\begin{array}{c} \varepsilon =T\times f_{s}\text{,} \end{array}$$

where *T* is the sampling period of a PPG signal and *f*_*s*_ is the sampling frequency of a PPG sensor.

As the refractory period of our heart is approximately 0.3 s [45], we set the difference between the start times of the two collected PPG signals to be no greater than this threshold; that is, the two PPG signals are considered to be synchronous, that is, the algorithm completes the time calibration. Therefore, we can get the time calibration formula as follows:

(2) $$\begin{array}{c} \left|\text{timestamp}\_\text{start}{\left(\tau \right)}_{1}-\text{timestamp}\_\text{start}{\left(\tau \right)}_{2}\right|\leq 3\text{.} \end{array}$$

Next, if the timestamps of the start and end of a PPG signal satisfy the following formula, it is considered that our proposed method in this paper can start and perform denoising. So, the execution turn-on condition is given by

(3) $$\begin{array}{c} \left|\text{timestamp}\_\text{start}{\left(\tau \right)}_{\text{soc}}-\text{timestamp}\_\text{end}{\left(\lambda \right)}_{\text{soc}}\right|\leq T\text{.} \end{array}$$

#### 3.3.2. Denoising Using Daubechies 5 Wavelet Transform

Denoising is done to reduce the influence of noise which is mainly generated by respiration and coupling circuits. For the preprocessing stage, we do not remove any more information from the raw PPG signals aside from reducing baseline wander and some low spike pulses in order to conveniently use the PPG signals in a follow-up stage.

The raw PPG signal is a time-seriesPPG={ppg(*m*)_soc_|m ∈ *ℕ*^*∗*^}, which is a composite signal consisting of major PPG information mppg(*m*), power interference pi(*m*), baseline wander *bw*(*m*), and other interference components ic(*m*). According to previous research [19], we introduce an additive function to describe the raw PPG signals, which can be described as follows:

(4) $$\begin{array}{c} \text{ppg}{\left(m\right)}_{\text{soc}}=\text{mppg}{\left(m\right)}_{\text{soc}}+\text{pi}{\left(m\right)}_{\text{soc}}+\text{bw}{\left(m\right)}_{\text{soc}}+\text{ic}{\left(m\right)}_{\text{soc}}\text{,} \end{array}$$

where *m* is any sample index of the PPG signals. When soc=1, ppg(m)_1_ indicates the left PPG signals; when soc=2, ppg(m)_2_ indicates the right PPG signals.

A Daubechies 5 (DB5) wavelet transform is applied to eliminating power interference and baseline wander components. The DB5 decomposition and reconstruction are used to deal with the raw PPG signal. The raw PPG is decomposed into 8-layer signals (0 to 7 layers), and we can observe that the 0 to 4 layers high-frequency component and the 7th-layer low frequency component are corrupted distinctly. Hence, we set a soft threshold in the 0 to 4 layers of high-frequency components to remove power interference and set the 7th-layer of low frequency component as 0. Finally, we perform wavelet reconstruction to obtain a new signal. Then, we get two noise-reduced signals in the following equation:

(5) $$\begin{array}{c} \text{ppg}{\left(m\right)}_{\text{soc}}=\text{mppg}{\left(m\right)}_{\text{soc}}+\text{ic}{\left(m\right)}_{soc}\text{,} \end{array}$$

where ic(*m*)_soc_ is mainly formed by various biological and motion artifacts. Our method does not need to solve motion artifacts and has an ability to locate the peak from the PPG signals with a small amount of motion artifacts.

### 3.4. Self-Iteration RR Interval Calculation

In this section, we describe the method of the self-iteration RR interval calculation in detail. This stage is one of the key steps to our method. According to the frequency feature of each PPG signal, the self-iteration RR interval calculation identifies automatically the systolic peak, preliminarily surmounting the impact of the BAs. In the process of this operation, no any threshold is set. The stage consists of three parts: self-iteration time window estimation, systolic peak identification in time domain PPG signal, and RR interval computation.

#### 3.4.1. Self-Iteration Window Estimation

We combine fast Fourier transform (FFT) and Nyquist theorem to derive the time window, also named as a self-iterative time window, which is utilized to detect the peak in every cardiac cycle, and this time window size is shorter than RR interval or cardiac cycle. First, according to FFT result, we confirm the maximum peak of PPG signal in frequency domain. We then get a transformation formula from Nyquist theorem and FFT frequency division theory. Finally, the self-iterative time window is deduced by importing the Nyquist transformation formula and PPG frequency domain maximum peak. This formula can be used to compute time window size directly. In the following statements, we expound our method.

FFT provides a signal transformation function from the time domain to the frequency domain. As shown in Figure 1, it is a frequency signal of a person under sitting conditions. Typically, the PPG signal frequency of a common person ranges from 0 Hz to 10 Hz. A 1-order difference is introduced to compute the peak. We get 24 peaks in Figure 1. These peaks comprise a candidate peak scope. In this scope, we only need the maximum peak (see peak P1 in Figure 4), which indicates the highest power point in the corresponding time domain point. It is convenient for us to locate the maximum peak *f*_max_ via the following formula. This is a simply processing and we can acquire one of the crucial parameters for the window estimation. The FFT peak search formula is given as follows:

(6) $$\begin{array}{c} f_{\max}=\max\;\left(f_{1},f_{2},f_{3},\ldots ,f_{n}\right),n=1,2,3,\ldots ,N\text{,} \end{array}$$

where *N* is the number of signal sampling points and *n* is frequency sequence number.

Nyquist theorem indicates that the theorem can be applied to a series of signal having a Fourier transform. After the FFT processing, the PPG signal conforms to Nyquist theory. On the grounds of sampling rate *f*_*s*_ and sampling quantity N, the sampling frequency *f*_*s*_ is divided into *N* parts based on *f*_*s*_/*N*. Then, we can get the PPG signal frequency expression *f*_*n*_ as follows:

(7) $$\begin{array}{c} f_{n}=\frac{\left(n-1\right)\times f_{s}}{N}\text{.} \end{array}$$

Then, we can get

(8) $$\begin{array}{c} n=\frac{f_{n}\times N}{f_{s}}+1\text{.} \end{array}$$

We introduce the maximum peak frequency into our formula. The variable *f*_*n*_ of equation (8) can be replaced by *f*_max_, we obtain a new equation of highest frequency sequence number *n*_max_ as follows:

(9) $$\begin{array}{c} n_{\max}=\frac{f_{\max}\times N}{f_{s}}+1\text{.} \end{array}$$

The highest frequency reflects peak information in per time domain cycle. Even if there are intense artifacts in different PPG signal cycles, it is hard for the highest power position to be changed. Because these artifacts commonly overlap with the peak, there is an increase in peak frequency. Its inclusion into computation is a befitting expression. Hence, the self-iteration window size *ω* is given by

(10) $$\begin{array}{c} \omega =g\left(N,f_{s},f_{\max}\right)\\ =\frac{N}{n_{\max}}\\ =\frac{f_{s}\times N}{f_{\max}\times N+f_{s}}\text{.} \end{array}$$

To facilitate iteration, we improve equation (10). During the next part, we adjust the coefficient of the self-iterative window size to complete iteration processing. When *α* ∈ [0,1], the improvement of equation (10) is defined as follows:

(11) $$\begin{array}{c} \omega^{\prime }=\left(1+\alpha \right)\times g\left(N,f_{s},f_{\max}\right)\\ =\left(1+\alpha \right)\times \frac{N}{n_{\max}}\\ =\left(1+\alpha \right)\times \frac{f_{s}\times N}{f_{\max}\times N+f_{s}}\text{.} \end{array}$$

#### 3.4.2. Systolic Peak Identification

In the light of peaks distribution features, we design and present a systolic peak identification method (SPIM) to measure the systolic peak. SPIM is a fusion technique which combines iterative thought and physiological characteristic. The basic idea of SPIM is that peak quantity is used as the iteration condition of SPIM. According to equation (11), SPIM enlarges the iteration window size by changing the iteration coefficient *α*. Because of the diversity of beat-to-beat intervals and vascular variability, the iteration window size carries systolic and diastolic information. Meanwhile, the peak number can embody the heart characteristic of the body, including vasculopathy, arrhythmias, and blood viscosity. As illustrated in Figure 5, SPIM is divided into six highlights in the following:

(1) *Peak Computing*. Any fixed threshold is not adopted to locate peak by SPIM. Using the following formulas, SPIM extracts all of the peaks in the sampling period. These peaks just are local maximum values. In this range, the following step of SPIM refines these local maximum values to find the systolic peak in each cardiac cycle. Formulas (12) and (13) are given as follows:
  (12) $$\begin{array}{c} ∆\text{ppg}{\left(m\right)}_{\text{soc}}=\text{ppg}{\left(m+1\right)}_{\text{soc}}-\text{ppg}{\left(m\right)}_{\text{soc}}\text{,} \end{array}$$
  (13) $$\begin{array}{c} \left\{\begin{array}{l} ∆\text{ppg}{\left(m-1\right)}_{\text{soc}}\geq 0\text{,}\\ ∆\text{ppg}{\left(m\right)}_{\text{soc}}<0\text{,}\\ \forall m\in N^{*}\text{,} \end{array}\right. \end{array}$$
where ∆ppg(*m*)_soc_ is the first-order backward difference. When equation (12) satisfies the constraint condition of equation (13), the corresponding ppg(*m*)_soc_ is the peak that we want to calculate. Let *u*(*r*), ∀*r* ∈ *ℕ*^*∗*^, be the peak, and then, the expression of the peak can be updated as follows:
  (14) $$\begin{array}{c} u{\left(r\right)}_{\text{soc}}∼\text{ppg}{\left(m\right)}_{\text{soc}}\text{,}\\ \text{iff}\left\{\begin{array}{l} ∆\text{ppg}{\left(m-1\right)}_{\text{soc}}\geq 0\text{,}\\ ∆\text{ppg}{\left(m\right)}_{\text{soc}}<0\text{,}\\ \forall m\in N^{*}\text{,}\\ \forall r\in \left[1,m\right]\text{,} \end{array}\right. \end{array}$$
where *m* is the corresponding sample index of peak on the PPG signals and *r* denotes the corresponding retrieval value of the peak. A peak set U consists of total peaks in all PPG signal recordings and is expressed as follows:
  (15) $$\begin{array}{c} U=\left\{u{\left(1\right)}_{\text{soc}},u{\left(2\right)}_{\text{soc}},u{\left(3\right)}_{\text{soc}},\ldots ,u{\left(\varphi \right)}_{\text{soc}}\right\},\varphi \in \left[1,r\right]\text{.} \end{array}$$
(2) Searching the highest peak in the current time window SPIM uses a difference comparison to search the highest peak in the scope of each time window. However, the highest peak in the initial time window is not the systolic peak and may be any peak. This peak does not take part in the computing of RR intervals.
(3) *Iterative Condition Judgment*. Except for the initial time window, the iterative condition judgment is executed in each time window. In the current time window, the number of peaks is treated as the iterative condition of adjusting the time window size. If the peak number *ϑ* is less than 3 in the current time window, the iteration coefficient *ϑ* is adjusted by SPIM at the step size of 0.1 until the peak quantity exceeds three points.
(4) *Identifying the Systolic Peak*. The highest peak, aside from the first highest one in the initial time window scope, is detected as the systolic peak. So, a data collection of the identified systolic peak U′ can be represented by
  (16) $$\begin{array}{c} U^{\prime }=\left\{u{\left(1\right)}_{\text{soc}}^{\prime },u{\left(2\right)}_{\text{soc}}^{\prime },u{\left(3\right)}_{\text{soc}}^{\prime },\ldots ,u{\left(\upsilon \right)}_{\text{soc}}^{\prime }\right\},\upsilon \in \left[1,\varphi \right]\text{.} \end{array}$$
That is to say that the next iteration time window starts with the prior systolic peak, and this peak does not participate in the next cycle iteration condition judgment.
(5) *Ending Condition.* If the peak number *υ* satisfies the condition *υ* ≤ 1 and *α*=0.2, then the SPIM considers that the process of systolic peak identification is over.

The fundamental reason for these steps is that a smooth PPG signal, which has few pulse spikes, is received after preprocessing. The remaining components comprise the main physiological information, such as systolic peak, diastolic peak, and other peaks.

#### 3.4.3. RR Interval Computation

In order to compute HR accurately, the EeHRA needs to have the ability to capture a precise RR interval. The RR interval is a significant cardiac manifestation, which reflects heart systolic and diastolic activity, and is made up of systolic and diastolic phases. Therefore, RR intervals can provide numerous types of physiologic information, especially HR computation and estimation.

In previous research, some literatures have demonstrated that RR interval can be measured from the ECG signals and PPG signals [46]. There are many effective approaches for calculating HR in some wearable devices via diverse models. Using time domain and frequency domain methods, both can get HR from PPG signals conveniently. In this paper, we calculate HR in time domain, and this approach facilitates HRV computing, IHR, and real-time application and can also provide more parameters (such as RR interval) than getting HR in the frequency domain.

For RR interval computation, we can define a time parameter *t*(*υ*)′, which is the time of corresponding to the peak *u*(*υ*)′. A PPG data collection interval [*W*_*a*_, *W*_*b*_] can be given based on reference [47]; thus, we get *u*(*υ*)′ ∈ [*W*_*a*_, *W*_*b*_]. The RR interval fundamental formula at time *s* can be computed as follows:

(17) $$\begin{array}{c} \text{RR}{\left(\upsilon \right)}_{\text{soc}}=\text{diff}\left(t{\left(\upsilon \right)}_{\text{soc}}^{\prime }\right)={t\left(\upsilon +1\right)}_{\text{soc}}^{\prime }-{t\left(\upsilon \right)}_{\text{soc}}^{\prime }\text{,} \end{array}$$

where the unit is second (*s*).

### 3.5. Heart Rate Pool Establishment and Abnormal Instantaneous Heart Rate Removal

In this section, we describe the establishment of heart rate pool (HRP), which provides the raw IHR data for the average HR estimation. However, the raw IHR data in the HRP include some abnormal data, which may be caused by the accumulated error of the previous calculation or may be caused by the BAs. Then, we introduce an unsupervised method to remove abnormal IHR, considering the contextual IHR relationship in the HRP. The computation flowchart of this section is as shown in Figure 6.

#### 3.5.1. HRP Establishment

The HRP is composed of IHR derived from multisensor PPG signals and provides computing and storage of IHR data. Each current IHR data entering the HRP not only can affect the calculation of the subsequent IHR data but also can be affected by the surrounding IHR data. Note that, in this paper, the multisensor PPG signals specifically mean that the two PPG signals are synchronously recorded by the two independent IoMT devices from two symmetric wrist areas on both sides of a body.

After the self-adaptive RR interval calculation, the EeHRA outputs the RR interval results in every cardiac cycle. According to literature [42], the HR estimation method in the time domain needs to use the RR interval to complete the computing function. In the sampling period, this allows an IHR value to be computed as follows:

(18) $$\begin{array}{c} \text{IHR}{\left(\upsilon \right)}_{\text{soc}}=\frac{60}{\text{RR}{\left(\upsilon \right)}_{\text{soc}}}\text{.} \end{array}$$

#### 3.5.2. Abnormal IHR Removal

The abnormal HR removal is a partition of the proposed method, which has a strong data filter function in the data domain to clean the data of the HRP instead of traditional preprocessing at the signal level. In the HRP, an abnormal IHR may come from heart rate variability (HRV), calculation bias of RR interval, or presence of BAs.

For abnormal IHR, it not only needs to be judged by its neighborhood samples but also needs to be judged by combining the neighborhood of its neighborhood samples. The main physiological reason for this is that the IHR does not undergo large change in a short period of time [26]. According to these features, we introduce an unsupervised outlier-detection method, AntiHubs [48], to remove the abnormal IHR from the HRP. The most important problem solved by this algorithm is to consider the neighborhood of the samples and the neighborhood of its neighborhood samples to find abnormal data. This is very consistent with the characteristics of the IHR data.

Before we describe the Antihubs (note that we just use the AntiHub2 in the reference) [48], two definitions should be given as follows.

**Definition 1 .**

(*k* − occurrences, Radovanović [48]). Given a finite set *H* ∈ *ℝ*^*d*^ of *h* samples, a distance, or similarity measure, the number of *k* − occurrences, indicated as *M*_*k*_(*x*), is the times *x* which means the number of occurrences in the *k* nearest neighbors of all other samples in *H*.

**Definition 2 .**

(*k* − occurrences, Radovanović [48]). For ∈(0,1), Hubs are the ⌈*gq*⌉ samples *x* ∈ *H* that have the highest values of *M*_*k*_(*x*). On the contrary, for ∈(0,1), *p* < 1 − *q*, AntiHubs are the ⌈*gq*⌉ samples *x* ∈ *H* that have the lowest values of *M*_*k*_(*x*).

To explore abnormal IHR, the k-occurrences of the sample *x*_*i*_, *M*_*k*_(*x*) and the *k* − occurrences of the neighborhood of *x*_*i*_, *M*_*k*_(*xj*), should be computed. Then, we need to compute a parameter *β*, which maximize the discrimination of *ξ*_*i*_. *ξ*_*i*_ can be given by

(19) $$\begin{array}{c} \xi_{i}=\left(1-\beta \right)\times M_{k}\left(x\right)+\beta \times \underset{x^{j}\in KNN\left(x\right)}{\sum }M_{k}\left(x\right)\text{.} \end{array}$$

Finally, we can get the score of the sample *x*_*i*_ by using the following equation:

(20) $$\begin{array}{c} \eta_{i}=1-\frac{1}{\xi_{i}+1}\text{,} \end{array}$$

where the higher the score *η*_*i*_ is, the more the sample *x*_*i*_ is considered an abnormal IHR. *η*_*i*_ ∈ (0,1]. For more details, please refer to the publishment of Radovanović [48].

### 3.6. Heart Rate Estimation

After section III-D, the HRP has minimized the number of IHRs that is affected by the algorithm iteration error and BAs, and the remaining IHRs are considered to be the IHRs that correctly reflect the HR components. Therefore, the final average HR estimation over the sampling period can be given by

(21) $$\begin{array}{c} \bar{\text{HR}}=\frac{\sum_{s=1}^{N}{\text{IHR}}_{1}\left(s\right)+\sum_{z=1}^{N}{\text{IHR}}_{2}\left(z\right)}{s+z}\text{.} \end{array}$$

## 4. Experimental Results and Performance Analysis

### 4.1. Experiment Setup

To verify our approach, a dataset is built with bilateral PPG signals and ECG reference signals. In this dataset, twenty-four measurements are performed on 12 subjects (9 males and 3 females, age from 24 to 54). Each subject is measured twice. Each measurement is divided into two phases. The first one is an adjustment stage for 30 s, followed by the data collection stage for 30 s, i.e., the sampling period of PPG signals is 30 s.

For increasing the complexity of the collected PPG signals during the experiment, we introduce the following two aspects. First, four of them have cardiovascular disease in different degrees, such as lightweight cardiopathy (subject 7) and hypertension (subject 2, 3, and 11). Others are healthy. Second, we adopt two different arm postures to collect PPG signals. During the experiment, the subjects just keep sitting to minimize arm movement. The both arms of subjects bend upward in the first measurement, and these of subject sags naturally in the second measurement. These signals are divided into three groups, the details of which are shown in Table 2.

In our experiment, two PPG signals are recorded from the double-sided wrists by two identical types of IoMT devices. Simultaneously, a commercial ECG device with dual electrodes is used to collect ECG signals from the chest. Three simultaneous signals are collected: two PPG signals as the measurement signals and the ECG signals as the gold standard signal. The ground truth of HR is computed from the gold standard ECG signals. We manually pick the R-peak in each cardio cycle for the purpose of restraining the detection errors.

### 4.2. Evaluation Metrics

To evaluate and quantify the performance of the proposed algorithm, we use three criterions to assess the consistency, accuracy, and computation time of our method. These three metrics can evaluate our method in different aspects.

As a standard index of consistency between the estimate value and ground truth value, the Bland–Altman plot is induced, which can describe the difference between every ground truth and corresponding to estimates. The limit of agreement is defined as [*μ* − 1.96 *δ*, *μ* +1.96 *δ*] in this part, *μ* is the average difference, and *δ* is the standard deviation.

For the accuracy of our proposed algorithm, the average absolute error percentage (AAEP) is an effective metric. It can be given as follows:

(22) $$\begin{array}{c} \text{AAEP}=\frac{1}{\psi }\overset{\psi }{\underset{l=1}{\sum }}\frac{\left|{\text{HR}}_{\text{true}}\left(l\right)-{\text{HR}}_{\text{est}}\left(l\right)\right|}{{\text{HR}}_{\text{true}}\left(l\right)}\text{.} \end{array}$$

In order to evaluate the low-latency computing capability of the our algorithm, we harness the total computation time of our proposed algorithm as the evaluation metric, which includes Bluetooth transmission time (*T*_1_), collection node execution time (*T*_2_), WIFI transmission time (*T*_3_), and computing node execution time (*T*_4_).

(23) $$\begin{array}{c} T_{\text{total}}=T_{1}+T_{2}+T_{3}+T_{4}\text{.} \end{array}$$

### 4.3. Results and Analysis

#### 4.3.1. Validation of HR Estimation Consistency

In order to evaluate the performance of HR estimation with multiple PPG signals in the case of complex peak distribution, Bland–Altman analysis is used in this paper to evaluate the consistency between the estimated value obtained by the proposed algorithm and the ground truth HR. It is worth noting that in order to allow Bland–Altman analysis to better evaluate our proposed method, we calculate the average HR every 15 seconds in this section.

As shown in Figure 7, it shows three Bland–Altman plots of HR estimation using the left PPG signals, right PPG signals, and bilateral PPG signals, respectively. The limit of agreement (LoA) of the EeHRA is (−10.67, 6.84) when comparing the estimated HR from the left PPG signals to the ground true HR from the gold standard ECG signals (see Figure 7(a)). The smaller range of LoA for the EeHRA using the right PPG signals is obtained (see Figure 7(b)), and the LoA is (−5.51, 7.01]). When using bilateral PPG signals, the LoA of the EeHRA is reduced to (−7.15, 5.82) (see Figure 7(c)). Apparently, the LoA of the EeHRA-bilateral has a similar range to that of the EeHRA-right; the LoA of the EeHRA-left has a greater range. This means that the EeHRA-bilateral method improves HR estimation results by using bilateral PPG signals. These results fully demonstrate the role of HRP and anomaly IHR detection in our proposed algorithm, removing some anomalous IHR and improving the accuracy of the algorithm. Furthermore, it also demonstrates that the possibility of large errors is less than that of the other two methods. For example, there are some large difference values in Figures 7(a) and 7(b). These difference values even are more than 5 bpm. However, the EeHRA using bilateral PPG signals removes these influences shown in Figure 7(c). Compared with using a single PPG signal, it is more effective for the EeHRA by using bilateral PPG signals to compute HR. In addition, for the EeHRA-bilateral method, there are 95.8% points within the LoA. Moreover, the LoA (−7.15, 5.82) can be accepted in the practical measurement. When using the left PPG signals and right PPG signals, there are 89.6% and 93.8% points within the corresponding to LoA, respectively. There are more unavailable HR values for these two cases than in the case of bilateral PPG signals. These results are statistically unacceptable.

Finally, for the case of bilateral PPG signals, the Bland–Altman analysis results of our method are all better than those of the methods using the left and right PPG signals. This is mainly due to the fusional property of the EeHRA, which enables it to fuse and extract effective HR information from bilateral PPG signals. This indicates that the EeHRA-bilateral using bilateral PPG signals overcomes the two other methods using a single PPG signal. Hence, the proposed method using bilateral PPG signals exceeds the two cases using a single PPG case in consistency.

#### 4.3.2. Accuracy Evaluation of HR Estimation

To explore the accuracy of the proposed algorithm, we use the average absolute error percentage (AAEP) to assess the proposed method on the dataset with three test groups, which can be seen in Table 2.  Figure 8 shows that the comparative results of the EeHRA-left, EeHRA-right, and EeHRA-bilateral method. The horizontal axis in Figure 8 represents the subjects; the vertical axis is the mean of absolute error percentages (MAEPs) of the two measurements for each subject, whose unit is %.

As shown in Figure 8, it is remarkable that most subjects' results have the presence of the BAs, some of which have a higher MAEP in the results of the EeHRA-left whilst the others show that the results of the EeHRA-right are higher than those of EeHRA-left. In most cases, the MAEP for EeHRA-bilateral is lower than that of one of EeHRA-left and EeHRA-right results, except for the results of subject 5. The AAEP result of the EeHRA-bilateral for all subjects is 4.14%. However, for all subjects, the AAEP of EeHRA-left and EeHRA-right is 4.79% and 4.40%, respectively. These results are 0.65% and 0.26% bigger than that of the EeHRA-bilateral. From the example of subjects 2, 3, 7, and 11, it is found that there are huge differences between the results of EeHRA-left and EeHRA-right. Nevertheless, the EeHRA can select some better IHR results from bilateral PPG signals to overcome the influence of the BAs and obtains a more accurate and consistent HR estimation. This immediately shows that the EeHRA-bilateral method improves the results of the EeHRA-left and EeHRA-right methods.

To sum up, we can see that our proposed method can overcome the BAs for different subjects and gets a better accurate HR result when using bilateral PPG signals than using a single PPG signal. Hence, the performance of EeHRA using bilateral PPG signals is better than that of EeHRA using a single PPG signal.

#### 4.3.3. Computation Time Analysis

Computation time is an important indicator for evaluating the low-latency properties of an edge computing-based healthcare application. In this paper, computation time is defined as the time interval required to transmit PPG signals across the edge network to the edge computing nodes and obtain the results of HR estimation. This interval includes Bluetooth transmission time, WIFI transmission time, collection node execution time, and computing node execution time.

In general, the performance of computation time is not only related to the complexity of the algorithm itself and calculation strategies but also to some other variables, such as the signal sampling rate, the length of the loaded data, and the configuration of the computing platforms. Therefore, in order to intuitively compare our proposed method with some existing methods on the HR estimation tasks, in terms of computation time, as shown in Table 3, we briefly organize and compare the representative HR estimation methods for recent years in this paper.

For the algorithms in references [17, 21], they obtain an excellent performance of HR estimation during intensive motion, using PPG signals captured by a wearable device. A significant advancement in the results of HR estimation can be achieved. We can see that although the method proposed by Zhang et al. used a high-performance personal computer (PC), it also takes about 3.5 h to process 3600 s PPG signals. Under the same sampling rate and data length, Khan et al. proposed a two-stage framework that improves the computation speed to 668 s and maintains good calculation accuracy. In spite of advances in computing speed, the complexity of these algorithms makes it difficult to port to the resource-constrained computing platforms such as edge devices and wearable devices. Han et al. [45] proposed an excellent work to accurately identify HR during sinus rhythm and cardiac arrhythmia. This work not only gets rid of the dependence on the acceleration signals but also enlarges the measurement condition of HR and provides a real-time detection capacity for estimating HR. It only takes 0.15 s to process a 30 s PPG signal on a PC to get a result of HR estimate, as shown in Table 3. In view of processing a 30 s PPG signal, the algorithm from Han et al. has the fastest computation speed. Unfortunately, this method is not available for edge devices or wearable devices. Furthermore, Burrello et al. [49] proposed a deep temporal convolutional network that is generated by a space exploration methodology, reducing motion artifacts, and computing HR. On an embedded device, as illustrated in Table 3, it takes 1.27 s to process 3 s PPG signals sampled at 100 Hz. However, this approach does not focus on the problem of accessing multiple PPG sensors to the edge network, but only for wearable-class devices.

In order to provide low-latency HR computing capabilities for multiple PPG sensors, we use three edge devices to form an edge network and test the computation time of our proposed method on different edge devices with hardware configurations, for example, Raspberry Pi 3B+ and Raspberry Pi 4B. As shown in Table 3, the computation time obtained by our method is 15.25 s on Raspberry Pi 3B+. By using Raspberry Pi 4B, an edge device with better hardware configuration, we obtain a better result with a computation time of 4.24 s. It is worth noting that our computation time results include the whole communication cost in the edge network for the 30 s of data, not just the algorithm computation time. We can find that, compared to the methods in references [17, 21] and reference [45], our proposed method has good low-latency performance on an edge computing platform with limited resources, without requiring the support of high-performance computing platforms.

## 5. Conclusion

In this paper, we present an edge-enabled HR estimation using multisensor PPG signals on the designed edge network. To the best of our knowledge, there are no frameworks or methods deployed on an edge network that process multisensor PPG signals and reach an acceptable performance in low-latency and accuracy. We separately introduce the PPG signal inherent frequency feature and an unsupervised anomaly detection method to mitigate the influence of BAs on HR estimation as much as possible, under the condition of multiple PPG signals. Furthermore, our method is designed and developed for edge networks and leverages the computing and low-latency communication ability of edge networks to provide computational support for heart rate estimation from multisensors PPG signals. Experimental results demonstrate the ability to compute HR with an accuracy and low-latency performance. In the future, our proposed method is expected to facilitate pervasive cardiovascular health monitoring and fitness management in the IoMT field.

## Figures and Tables

**Figure 1:** An example of the biological artifacts (BAs). There is a vascular lesion in the left vascular branch. The dicrotic notch and diastolic peak in the left PPG signals (blue line) have almost disappeared. In contrast, the right PPG signals (pink line) is well.

**Figure 2:** Overview of the edge-enabled heart rate estimation approach. Red PPG signals and blue PPG signals are collected from the right and left wrist regions, respectively. ECG signals as reference signals are gathered from the chest synchronously. In the HRP, a red circle represents an HR value derived from the right PPG signals. Similarly, a blue circle means an HR measured from the left PPG signals. Four edge nodes are used in our approach.

**Figure 3:** A scheme for real-world edge network with four resource-constrained devices.

**Figure 4:** Frequency domain waveform of a PPG signal. Horizontal axis means frequency of a PPG signal. Red star shows peak chosen by us.

**Figure 5:** SPIM processing for two random recorded PPG signals.

**Figure 6:** The computation procedure of the HRP, which includes two major components: establishing HRP and abnormal IHR removal. In the panel bottom, we show the raw PPG signals and the computation of RR intervals and IHRs. In the PPG signals layer, the blue signals are collected from the left wrist area. Similarly, the red one is the right wrist PPG signals. RR interval and IHR in each cardiac cycle are in one-to-one correspondence. All the IHR results constitute an HRP.

**Figure 7:** Bland–Altman plots. (a) Results of left PPG signals. (b) Results of right PPG signals. (c) Results of bilateral PPG signals. All results are compared with the ground truth value derived from the ECG signals.

**Figure 8:** The mean of the absolute error percentage (MAEP) for two measurements of our method.

**Table 1:** A research review of artifact removal techniques based on PPG sensors in recent years.

Published works	Activities	PPG sensor wavelength	PPG sensor quantity and deployment area	Artifact types	Algorithm types	Reference sensors
Zhang [17]	HR	PPG (515 nm, green)	1 Wrist	MA	JOSS	Accelerometer
Jarchi and Casson [18]	IHR	PPG (515 nm, green)	1 Wrist	MA	SMA	Accelerometer
Wijshoff et al. [19]	PR,IBI, S_p_O_2_	PPG (660 nm, red; 900 nm, near infrared)	2 Forehead	BMA + RMA	LMS	Accelerometer + laser diode
Lee et al. [20]	HR	PPG (570 nm, green)	9 Wrist	MA	SVD	PPG
Khan et al. [21]	HR	PPG (515 nm, green)	1-2 Wrist	MA + BA	RLS	Accelerometer
Dao et al. [22]	HR, S_p_O_2_	PPG (940 nm, infrared)	2 Forehead or finger	MA	VFCDM + SVM	None
Antink et al. [25]	RR interval	PPG (near infrared)	1 Back	MA	xCLIE	ECG, BCG, HFI, and camera
Warren et al. [27]	PR	PPG (660 nm, red; 940 nm, infrared)	4 Forehead	MA	MTM	Accelerometer + PPG (red and infrared)
Antink et al. [43]	HR	PPG (-, green)	1 Forehead	MA	Bayesian	ECG, BCG + webcam
Arunkumar and Bhaskar [44]	HR	PPG (515 nm, green)	2 Wrist	MA	RLS + NLMS + FFT + PV	Accelerometer
Liu et al. [4]	HR	rPPG	1 Face	MA	DFROIT + PCKF	ECG + BCG

*Note.* MA: motion artifacts; PR: pulse rate; BMA: body motion artifact; RMA: relative motion artifact; SVD: singular value decomposition; JOSS: joint sparse spectrum; VFCDM: variable frequency complex demodulation; SVM: support vector machine; ECG: electrocardiogram; BCG: ballistocardiogram; HFI: high-frequency impedance; xCLIE: multichannel extended continuous local interval estimator; PF: particle filter; ABP: arterial blood pressure; SFM: sensor fusion method; TBC: tree-based classifier; MDC: minimum-distance classifier; MTM: multichannel template matching; TM: threshold method; NLMS: normalized least mean squares; FFT: fast fourier transform; PV: phase vocoder; rPPG: remote photoplethysmography; DFROIT: deep facial ROI tracker; and PCKF: pose constrained Kalman filter.

**Table 2:** The three groups of PPG signals in detail.

Group nos.	Signal source	Number of signals	Sampling period (s)	Methods
1	Left wrist area	24	30	EeHRA-left^1^
2	Right wrist area	24	30	EeHRA-right^2^
3	Bilateral wrist areas	48	30	EeHRA-bilateral^3^

^1^EeHRA-left denotes that the EeHRA method uses the left PPG signals as the signal source. ^2^EeHRA-right denotes that the EeHRA method uses the right PPG signals as the signal source. ^3^EeHRA-bilateral denotes that the EeHRA method uses the bilateral PPG signals as the signal source.

**Table 3:** Comparison of our proposed method with several existing methods on computation time.

Nos.	Devices and methods	Signal type	Sampling rate (Hz)	Loading data length (s)	Processing platform configuration	Computation time
1	PC, Zhang [17]	PPG	125	3600	Intel Core-i7 4790 at 3.60 GHz, 8 GB RAM, windows 7 64 bit	3.5 h
2	PC, Khan et al. [21]	PPG	125	3600	Intel Core-i7 4790@3.60 GHz, 8 GB RAM, windows 7 64 bit	668 s
3	PC, Han et al. [45]	PPG	500	30	Intel Core i7 7700HQ@2.8 GHz, RAM 16.0 GB	0.15 s
4	Wearable device, Burrello et al. [49]	PPG	100	3	STM32H743ZIT6 with480 MHz, 1 MB RAM, and 2 MB FLASH	1.27 s
5	Edge device, our method	PPG	200	30	Raspberry Pi 3B+, ARM Cortex-A53@1.4 GHz 2 GB SDRAM	15.25 s
6	Edge device, our method	PPG	200	30	Raspberry Pi 4B, ARM Cortex-A72@1.5 GHz, 4 GB SDRAM	4.24 s

*Note.* There is a special case in this experiment, which aims at subjects 3 and 7. For the case of subject 3, the MAEP of the EeHRA-right method is more than that of the EeHRA-left and EeHRA-bilateral methods. For a similar situation, subject 7 gets the highest MAEP using the EeHRA-left. These problems result in higher MAEP of the EeHRA-bilateral method. Furthermore, in these situations, the abnormal IHR mechanism fails because the scores of some unuseful IHR values in the HRP are not close to 1. According to the principle of the AntIHub, these IHRs are deemed to be the normal data. So, in this condition, the MAEP of the EeHRA-bilateral increases.

## Data Availability

The data that support the findings of this study are available on request from the corresponding author.

## References

[1] Laila I., Arifin A., Armynah B. (2022). Internet of medical things (iomt)-based heart rate and body temperature monitoring system. *Indonesian Physical Review*.

[2] Niaz F., Khalid M., Ullah Z., Aslam N., Raza M., Priyan M. (2020). A bonded channel in cognitive wireless body area network based on ieee 802.15. 6 and internet of things. *Computer Communications*.

[3] Tiwari A., Liaqat S., Liaqat D., Gabel M., de Lara E., Falk T. H. Remote copd severity and exacerbation detection using heart rate and activity data measured from a wearable device.

[4] Liu Y., Qin B., Li R. (2021). Motion-robust multimodal heart rate estimation using bcg fused remote-ppg with deep facial roi tracker and pose constrained kalman filter. *IEEE Transactions on Instrumentation and Measurement*.

[5] Nemcova A., Jordanova I., Varecka M. (2020). Monitoring of heart rate, blood oxygen saturation, and blood pressure using a smartphone. *Biomedical Signal Processing and Control*.

[6] Shabaan M., Arshid K., Yaqub M. (2020). Survey: smartphone-based assessment of cardiovascular diseases using ecg and ppg analysis. *BMC Medical Informatics and Decision Making*.

[7] Lin X., Wu J., Mumtaz S., Garg S., Li J., Guizani M. (2021). Blockchain-basedon-demand computing resource trading in iov-assisted smart city. *IEEE Transactions on Emerging Topics in Computing*.

[8] Zrar Ghafoor K., Kong L., Zeadally S. (2020). Millimeter-wave communication for internet of vehicles: status, challenges, and perspectives. *IEEE Internet of Things Journal*.

[9] Jiang D., Wang F., Lv Z. (2023). Qoe-aware efficient content distribution scheme for satellite-terrestrial networks. *IEEE Transactions on Mobile Computing*.

[10] Lin S., Zheng B., Alexandropoulos G. C., Wen M., Chen F., Mumtaz S. (2020). Adaptive transmission for reconfigurable intelligent surface-assisted ofdm wireless communications. *IEEE Journal on Selected Areas in Communications*.

[11] Li Q., Chen Y., Zhang A. (2022). A Super-resolution Flexible Video Coding Solution for Improving Live Streaming Quality. *IEEE Transactions on Multimedia*.

[12] Zhang A., Li Q., Chen Y. (2021). Video super-resolution and caching–an edge-assisted adaptive video streaming solution. *IEEE Transactions on Broadcasting*.

[13] Ma X., Li Q., Zou L. (2022). Qava: Qoe-Aware Adaptive Video Bitrate Aggregation for Http Live Streaming Based on Smart Edge Computing. *IEEE Transactions on Broadcasting*.

[14] Wang H., Li Q., Sun H. (2023). Vabus: edge-cloudreal-time video analytics via background understanding and subtraction. *IEEE Journal on Selected Areas in Communications*.

[15] Kenner T. (2004). Biological asymmetry and cardiovascular blood transport. *Cardiovascular Engineering*.

[16] Wu J.-X., Li C.-M., Ho Y.-R., Wu M.-J., Huang P.-T., Lin C. H. (2016). Bilateral photoplethysmography analysis for peripheral arterial stenosis screening with a fractional-order integrator and info-gapdecision-making. *IEEE Sensors Journal*.

[17] Zhang Z. (2015). Photoplethysmography-based heart rate monitoring in physical activities via joint sparse spectrum reconstruction. *IEEE Transactions on Biomedical Engineering*.

[18] Jarchi D., Casson A. J. (2017). Towards photoplethysmography-based estimation of instantaneous heart rate during physical activity. *IEEE Transactions on Biomedical Engineering*.

[19] Wijshoff R. W. C. G. R., Mischi M., Aarts R. M. (2017). Reduction of periodic motion artifacts in photoplethysmography. *IEEE Transactions on Biomedical Engineering*.

[20] Lee H. W., Chung H., Ko H., Lee J. (2018). Wearable multichannel photoplethysmography framework for heart rate monitoring during intensive exercise. *IEEE Sensors Journal*.

[21] Khan E., Al Hossain F., Uddin S. Z., Alam S. K., Hasan M. K. (2016). A robust heart rate monitoring scheme using photoplethysmographic signals corrupted by intense motion artifacts. *IEEE Transactions on Biomedical Engineering*.

[22] Dao D., Salehizadeh S. M. A., Noh Y. (2017). A robust motion artifact detection algorithm for accurate detection of heart rates from photoplethysmographic signals using time–frequency spectral features. *IEEE Journal of Biomedical and Health Informatics*.

[23] Chowdhury S. S., Hyder R., Hafiz M. S. B., Haque M. A. (2018). Real-time robust heart rate estimation from wrist-type ppg signals using multiple reference adaptive noise cancellation. *IEEE Journal of Biomedical and Health Informatics*.

[24] Lin W.-J., Ma H.-P. A physiological information extraction method based on wearable ppg sensors with motion artifact removal.

[25] Antink C. H., Schulz F., Leonhardt S., Walter M. (2018). Motion artifact quantification and sensor fusion for unobtrusive health monitoring. *Sensors*.

[26] Nathan V., Jafari R. (2018). Particle filtering and sensor fusion for robust heart rate monitoring using wearable sensors. *IEEE Journal of Biomedical and Health Informatics*.

[27] Warren K., Harvey J. R., Chon K. H., Mendelson Y. (2016). Improving pulse rate measurements during random motion using a wearable multichannel reflectance photoplethysmograph. *Sensors*.

[28] Maeda Y., Sekine M., Tamura T. (2010). Relationship between measurement site and motion artifacts in wearable reflected photoplethysmography. *Journal of Medical Systems*.

[29] Sun Y., Liu J., Bashir A. K. (2021). E-Cis: Edge-Based Classifier Identification Scheme in green and Sustainable Iot Smart City. *Sustainable Cities and Society*.

[30] Tan L., Yu K., Bashir A. K. (2021). Toward Real-Time and Efficient Cardiovascular Monitoring for Covid-19 Patients by 5g-Enabled Wearable Medical Devices: A Deep Learning Approach. *Neural Computing and Applications*.

[31] Dassanayake P. M., Anjum A., Bashir A. K., Bacon J., Saleem R., Manning W. (2022). A deep learning based explainable control system for reconfigurable networks of edge devices. *IEEE Transactions on Network Science and Engineering*.

[32] Zhu F., Ning Y., Chen X., Zhao Y., Gang Y. (2021). On removing potential redundant constraints for svor learning. *Applied Soft Computing*.

[33] Zhu F., Gao J. Y., Yang J., Ye N. (2022). Neighborhood linear discriminant analysis. *Pattern Recognition*.

[34] Zhu F., Gao J., Xu C., Yang J., Tao D. (2018). On selecting effective patterns for fast support vector regression training. *IEEE Transactions on Neural Networks and Learning Systems*.

[35] Zheng H., Shi Z., Zhou C., Haardt M., Chen J. (2021). Coupled coarray tensor cpd for doa estimation with coprime l-shaped array. *IEEE Signal Processing Letters*.

[36] Zhou C., Gu Y., He S., Shi Z. (2018). A robust and efficient algorithm for coprime array adaptive beamforming. *IEEE Transactions on Vehicular Technology*.

[37] Zhou C., Gu Y., Shi Z., Zhang Y. D. (2018). Off-grid direction-of-arrival estimation using coprime array interpolation. *IEEE Signal Processing Letters*.

[38] Fischer C., Domer B., Wibmer T., Penzel T. (2017). An algorithm for real-time pulse waveform segmentation and artifact detection in photoplethysmograms. *IEEE Journal of Biomedical and Health Informatics*.

[39] Wu H.-T., Lee K.-W., Pan W.-Y., Liu A. B., Sun C.-K. (2017). Difference in bilateral digital volume pulse as a novel non-invasive approach to assessing arteriosclerosis in aged and diabetic subjects: a preliminary study. *Diabetes and Vascular Disease Research*.

[40] Budidha K., Kyriacou P. A. Investigation of pulse transit times utilizing multisite reflectance photoplethysmography under conditions of artificially induced peripheral vasoconstriction.

[41] Maria C. D., Sharkey E., Klinge A. Feasibility of monitoring vascular ageing by multi-site photoplethysmography.

[42] Clark C. E., Taylor R. S., Shore A. C., Campbell J. L. (2016). Prevalence of systolic inter-arm differences in blood pressure for different primary care populations: systematic review and meta-analysis. *British Journal of General Practice*.

[43] Antink C. H., Gao H., Brüser C., Leonhardt S. (2015). Beat-to-beat heart rate estimation fusing multimodal video and sensor data. *Biomedical Optics Express*.

[44] Arunkumar K. R., Bhaskar M. (2020). Robust de-noising technique for accurate heart rate estimation using wrist-type ppg signals. *IEEE Sensors Journal*.

[45] Han D., Bashar S. K., Lázaro J. (2022). A real-time ppg peak detection method for accurate determination of heart rate during sinus rhythm and cardiac arrhythmia. *Biosensors*.

[46] Grooby E., He J., Kiewsky J. (2021). Neonatal heart and lung sound quality assessment for robust heart and breathing rate estimation for telehealth applications. *IEEE Journal of Biomedical and Health Informatics*.

[47] Gee A. H., Barbieri R., Paydarfar D., Indic P. (2017). Predicting bradycardia in preterm infants using point process analysis of heart rate. *IEEE Transactions on Biomedical Engineering*.

[48] Radovanović M., Nanopoulos A., Ivanović M. (2015). Reverse nearest neighbors in unsupervised distance-based outlier detection. *IEEE Transactions on Knowledge and Data Engineering*.

[49] Burrello A., Pagliari D. J., Risso M. (2021). Q-ppg: energy-efficientppg-based heart rate monitoring on wearable devices. *IEEE Transactions on Biomedical Circuits and Systems*.

